The article "Analysis of the Relationship between Dance Action and Health Psychology in the Process of Dance Performance Teaching Environment" was retracted in 2023. Reasons: unreliable results or conclusions; concerns about the data; concerns about the results or conclusions; concerns about the peer review.

# Analysis of the Relationship between Dance Action and Health Psychology in the Process of Dance Performance Teaching Environment

**DOI:** 10.1155/2022/3830522

**Published:** 2022-09-14

**Authors:** Jing Huang

**Affiliations:** School of Music, Shanxi Datong University, Datong Shanxi 037009, China

## Abstract

One of the public fundamental disciplines that is typically put up among the professional teaching units in universities is dance. In order for this sports project with fitness, mental health, and aesthetic functions to be widely developed in universities, the use of reasonable, scientific, and targeted teaching methods can effectively improve the instructional effect. At the same time, it has further promoted the quality of education in universities and implemented the guiding ideology of “health first.” In order to avoid the classifier's performance-degrading effects brought on by the high dimension, this research suggests combining the classifier's psychological stress identification algorithm with a particle swarm optimization (PSO) approach. The experimental findings reveal that the PSO-SVM algorithm, PSO-BP algorithm, improved PSO-SVM algorithm, and improved PSO-BP algorithm, respectively, have recognition rates for psychological stress of 82.50%, 84.50%, 90.17%, and 94.83%. Additionally, the recognition rates of the improved PSO classifier are significantly higher than those of the basic PSO algorithm, demonstrating the improved PSO algorithm's strong generalization ability in optimization.

## 1. Introduction

With the introduction of western advanced ideas and industrial technology into China in the 19th century, it also brought different national cultures, among which ballroom dancing, the predecessor of sports dance, was one. This new dance was gradually accepted by the upper class and developed in China's coastal areas such as Shanghai, Guangzhou, and Tianjin [1]. In 1990, the first “National Sports Dance Championship” was held. The unique gentlemanly style and graceful dance of sports dance art, as well as the holding of large-scale competitions and the deepening exchanges between Chinese and foreign sports dance cultures, continued to promote the development of sports dance projects, which were loved by people of different cultural classes. Sports dance competitions, associations, and clubs all over the country mushroomed [2].

In the 21st century, sports dance has been known by more people, competitions of different sizes have emerged in an endless stream, and dance exchanges between China and foreign countries have become closer and closer. Chinese players have emerged in the international arena, demonstrating China's strength. People who study sports dance have developed from the middle-aged to the younger age, and more children and teenagers have become important people and reserve talents in sports dance learning [3]. Since then, most universities in China have set up special or public courses of sports dance, which has produced more athletes and dance teachers, but at the same time, many problems have emerged. Because dance teachers lack the understanding of dance theory and dance instructional mode and method in teaching, they only rely on “experience” to teach, which leads to a great discount on the effect of training talents [4].

With the development of network technology, network resources grow rapidly, and rich network information resources become an important source for people to obtain information [5]. However, while people are enjoying the convenience brought by information technology, how to accurately express the demand for network resources and how to accurately and effectively search for resources has become a major problem faced by network users [6]. Dance education is one of the effective ways to solve this problem. Dance education is a comprehensive art education activity organization and implementation form that simultaneously absorbs and integrates aesthetic education elements, moral education elements, and emotional education elements. In the process of teaching and training students of various majors in universities, dance education widely undertakes and plays the task of purifying students' minds, cultivating students' sentiments, and combining teaching with beauty [7]. In the process of organizing and carrying out the teaching work of dance art in universities, the teachers can take advantage of the rationalization of the introduction and arrangement of teaching contents and the rationalization of the design and implementation of the organization and implementation of teaching work. Supervise the students in universities to gradually build and form the ability to discover, feel, understand, and create beauty, guide and promote the majority of students in universities to consciously and actively build and form the consciousness of love and pursuit of beauty in the process of daily participation in learning and life, and then support and protect the moral concepts and artistic sentiments of the majority of students in universities, and spiritual quality can be improved and sublimated to a certain extent [8]. Dance is so close to the body, and the body is so close to us. In other words, we cannot leave our bodies for a moment; the body undertakes all the tasks that we need to meet our physiological needs. In order to successfully complete the task, the body has been developed by human beings to the highest comprehensive level in the life world at least today, but our perception of the body seems to be gradually blurred [9]. From this point of view alone, I do not know whether it is a retrogression of human civilization in the sense of “body consciousness”. Even if we create dance, it preserves the most active part of human body movements and emotions. It is based on body expression; the fundamental purpose is emotional communication [10].

According to psychological research, the assessment methods of psychological stress mainly include stress response questionnaire, life event resolution questionnaire, and perceived stress scale. Although these methods can roughly evaluate the educational psychological state of the tester, they are not accurate enough and have certain subjectivity. Nowadays, the collection and processing technology of physiological signals is more and more mature, and the physiological signals can effectively and accurately reflect the psychological stress state of the human body, and will not have too much impact on the tester. Therefore, it is an internationally recognized effective way to use physiological signals to evaluate stress. Therefore, in the teaching process, in addition to the conventional sports teaching methods, according to the characteristics of sports dance, scientific and targeted teaching methods should be adopted to improve the instructional effect, make up for the deficiencies in the above aspects, and further improve the sports dance theory, which has both practical and theoretical significance in sports dance teaching. In addition to constructing the support vector machine classification model and the SVM network model, this paper also introduces the particle swarm optimization algorithm. It trains and evaluates the classifiers using a particle swarm optimization approach combined with the two classifiers. This study enhances the particle swarm optimization (PSO) algorithm, adopts the particle swarm optimization model with contraction factor, ensures convergence of the PSO algorithm by choosing suitable parameters, and eliminates the speed boundary limit in order to increase the recognition rate of psychological stress. The SVM neural network and the support vector machine method are then optimized using the basic and advanced particle swarm optimization techniques in combination with the two classifiers, and the simulation results of the four algorithms are compared and examined.

## 2. Related Work

Most of the research of Chinese scholars on the instructional mode of dance sports in universities is based on experimental research and current situation analysis. They have not comprehensively analyzed and summarized the instructional mode of dance sports in universities and have not built a complete and stable instructional mode and framework according to the characteristics of the discipline. Therefore, this study hopes to play a role of guidance and reference. Constructing the instructional mode and framework of sports dance in universities plays an active role in improving the teaching theory of sports dance.

Bortnyk, based on the psychological and physiological characteristics of different groups and the macroteaching concept, qualitatively put forward the significance of heuristic and exploratory teaching methods in sports dance class and matched reasonable assessment methods to achieve the teaching objectives [11]. Jooste et al. pointed out that the appearance is also the mental image, but the name is different. In fact, the imagery in imagery training is a kind of generalized imagery, that is, mental phenomenon that includes imagination and is characterized by images [12]. The relevant outline issued by Sophy in 2018 advocates “taking students as the center, fully respecting students' dominant position in learning; taking teachers as the leading role, giving full play to teachers' guiding role; taking exploratory learning as the main mode, giving full play to open thinking habits; taking effectiveness as the basic principle, fully exploring the time and space of physical education courses [13]. According to Jin in the application research of multimedia CAI technology in physical education teaching, CAI technology was expounded and applied to physical education teaching, with obvious effect [14]. An and Mal-E combined the network course of “school dance” with the theory and made contributions to the comprehensive development of sports dance teaching. Many computer professionals have made contributions to the research of network teaching in the field of sports [15]. In the study of Kirsch, according to the current situation of dance teaching in universities, a set of long-distance online dance teaching system is designed, and a multicategory dance teaching system based on B/S network structure is realized. Based on the three roles of teachers, students, and administrators, an online teaching learning and offline-interactive instructional mode with a complete database are constructed, which enriches the diversity of teaching means and teaching methods in universities [16]. Orgs et al. pointed out that talent training, cultural inheritance and protection, and advanced concepts and methods in teaching constitute the core link of Chinese dance teaching and development. This is undoubtedly a summary of the teaching experience of Chinese dance in the past 20 years, and also points out the way forward for the future teaching focus and direction of dance [17]. Armstrong et al. proposed that sports dance, as a “foreign product,” is a dance that contains rich national culture. Each dance contains a unique national style and charm. Only by deeply understanding the cultural background of different nationalities can dancers better grasp the dance style. However, in the current sports dance education, most colleges and universities pay too much attention to the training of movement skills in the teaching of professional courses, neglecting the influence of the dance cultural atmosphere on the dancers' dance forms, resulting in the students' understanding and mastery of dance techniques only exist on the surface and in the form, and the dances they jump out always feel rigid and lack charm and connotation [18]. ASAF et al. put forward relevant countermeasures: first, optimize the structure of teachers and improve the professional quality of teachers; second, lay stress on the retraining of teachers after taking office, improve the scientific research level of teachers, and improve the teaching quality; third, increase sports dance competitions and academic exchanges among universities; fourth, standardize the teaching system of sports dance and build and improve the teaching theory, course content, and instructional mode of sports dance in universities [19]. Aiming at this practical research, Alexiadis and Daras conducted a small-scale aerobics network teaching experimental research on college education students. It was found in the experimental process that students are generally satisfied with the network course teaching [20].

## 3. Methodology

### 3.1. Analysis of Online Dance Teaching System

Since the new century, with the rapid and orderly development of China's contemporary social science and technology research, economic construction, and cultural construction, the talent factor has gradually become a representative factor to support and assist countries around the world to achieve rapid, stable, and orderly development, which indirectly poses a great challenge to the talent training mode of universities being applied in China. Since the goal of the dance teaching curriculum is to train students to learn dance knowledge and master dance skills, it is also a key course for dance students to exercise their temperament and shape good bodies. How to effectively use the rich teaching resources on the Internet is a key problem that needs to be solved at present. Judging from the basic memory decline curve of human brain, students may not remember exactly the same dance movements as the previous teacher's body language demonstration, so this will weaken the core significance of dance teaching. Every demonstration or lecture by a teacher will partially limit students' learning and knowledge infusion, but it is entirely possible to realize this appeal if computer technology is used. For example, teachers record each demonstration action into the website and show the dance through some three-dimensional action software or auxiliary instructional mode. First of all, this instructional mode can greatly facilitate students, and they can watch the teaching videos online anytime and anywhere; Dance explanation is the basic link of dance classroom teaching.

In the dance training class, the teacher's explanation work is divided into two parts. First, explain the essentials of movements comprehensively and accurately, which is the part of theoretical teaching. Second is to correct the shortcomings of dance movements in dance training, which is the part of practice teaching. In this learning stage, teachers' language foundation is particularly important. They can summarize the specific contents and essentials of movements in concise and accurate language, enhance students' interest in dance learning, and improve their own dance level. As a teacher majoring in dance, he or she has been engaged in dance education for many years, or he or she has been an actor with rich stage performance experience. He or she should be familiar with the background knowledge of the dance he or she teaches, and can also supplement it in many ways. During the teaching work, rich historical and cultural knowledge and vivid language can fully arouse students' interests and help them understand the real connotation of the dance content. That is to say, just like all teaching work, the main purpose is to cultivate talents, among which professional level and moral quality are equally important. Teachers practice and preach with rigorous language, so that students can experience a rigorous attitude towards learning. Explain and practice classroom discipline requirements in person. Students can listen to teachers' language, observe the emotions expressed by teachers' language, and understand teachers' requirements in the classroom. Over time, students will establish a correct attitude towards life, which will be of great benefit to students' dance learning and even their whole life. Of course, in this process, dance teachers are strict with their own behavior, which plays a good role in demonstrating and setting an example. The roles of each component of the system have been organized in accordance with the demand relationship among administrators, instructors, and students that was examined above.  Figure 1 depicts the functions of each submodule in the online dance instruction system.

Eight primary design tenets are covered by the online dance instruction system's design principles and goals: affordability, security, expansibility, progression, dependability, practicality, simplicity, and hierarchical modularity. Below, they are fully studied and expanded upon. The two common software architectures are C/S architecture and B/S architecture. Currently, the client/server architecture, often known as C/S (Client/Server), is one that is frequently used in software. The existing Internet's requirements, the trend of multiparty interconnection, global network opening, and information globalisation cannot be met by the classic C/S architecture, which is why the B/S architecture is progressively gaining popularity. When this architecture first appears, it challenges people's preconceived notions of conventional software architecture and offers software engineers a fresh perspective on their work. The architecture of the remote dance instruction system proposed in this paper is depicted in Figure 2.

Three blocks, the client, the network server, and the database server, make up the usual three-layer B/S physical structure in the architecture diagram of the remote dance instruction system illustrated in Figure 2. The client's primary focus is on determining whether the user's chosen browser's communication protocol and the back end server port are compatible. Different browsers will have different automatic firewall configurations. In addition, when configuring IIS protocol with the network server, they should take compatibility into account. For instance, the server contains four separate contents, including HTML, http://asp.net, JavaScript, and ADO Net, which is connected with the back-end database server while transmitting and receiving data through the HTTP protocol. It basically performs the following tasks: uploading the video resources for teachers' courseware, retrieving the list of teachers' uploaded resources, querying students' information, querying students' courses, and online learning and course selection.

### 3.2. PSO Feature Extraction Based Dance Psychoanalysis Algorithm

Dance psychological factors belong to a branch of psychological factors. It makes relevant exploration and research on psychological factors in dance performance and teaching, and provides theoretical basis and scientific basis for dance teaching. Information security with information hiding technology as its core technology is disguised information security. The difference between camouflage information security technology and traditional password technology is that password only hides the content of information, while information camouflage hides not only the content but also the existence of information. Camouflage information security technology provides a security mode different from encryption, and its security comes from the paralysis of the perception of the third party. In this process, the role of carrier information actually includes two aspects: (1) providing a channel for transmitting information; (2) Provide camouflage for the transmission of hidden information.

The interdisciplinary or marginal disciplines formed with various disciplines of psychology, such as cultural psychology, educational psychology, and sports psychology, are still new disciplines in China. Especially art psychology, dance psychology, performance psychology and so on, are all under construction. The so-called performance psychology refers to the sum of the behaviors and mental activities related to dance activities and their interactions. Singing psychology is a new discipline that studies the psychological phenomena and teaching practice of dance teachers, students, and all performers. It can help us deeply understand the internal relationship and objective laws between dance and brain thinking activities, so as to improve the teaching level of dance teachers, enhance students' learning ability and give full play to dancers' stage performance level.

Eberhart and Kennedy in the US proposed the PSO algorithm in 1995. It is an algorithm for optimization that mimics fish and birds. PSO's origins can be traced to the discovery, following observation of some animals' social behaviors, that animal groups' contributions to knowledge have evolutionary benefits. This algorithm was then built around this discovery. Although individual creatures in nature lack intelligence, the entire biological community is capable of solving challenging issues. PSO technique was initially employed to address continuous optimization issues. Artificial intelligence has now been applied to combinatorial optimization issues as a result of ongoing research in the field. It has been highly respected and extensively researched by academics since it not only preserves the original global search method but also has easy operation compared to genetic algorithms and can dynamically adapt the search circumstances of currently tracked particles.

The fitness value is first calculated, then the fitness function model is built, and finally an ideal solution is found by contrasting the fitness values of the individual particles. The best position among them is designated as Pbest_*i*_ = (Pbest_*i*1_, Pbest_*i*2_.Pbest_*i*3_, ⋯,Pbest_*iD*_)^*T*^, and by comparing every particle, we can determine the optimal position for the entire population. When the optimal solution is found, the next generation of particles can be calculated by formulas (1) and (2), and the search and calculation can be repeated until an optimal solution is obtained.

(1) $$\begin{array}{c} V_{i}^{n+1}=V_{i}^{n}+C_{1}\times {\mathrm{rand}}_{1}\left(\;\right)\times \left({\text{Pbest}}_{i}-X_{i}^{n}\right)+C_{2}{\mathrm{rand}}_{2}\left(\;\right)\times \left(\text{Gbest}-X_{i}^{n}\right), \end{array}$$

(2) $$\begin{array}{c} X_{i}^{n+1}=X_{i}^{n}+V_{i}^{n}. \end{array}$$

The steps and flow of particle swarm optimization are as follows: (1) initialize the particle swarm, and randomly set the initial position *X*_*i*_ and initial velocity *V*_*i*_ of each particle; (2) calculate the fitness value and evaluate the fitness of each particle; (3) update the individual optimum fitness value of each particle; (4) compare the current fitness value of each particle with the fitness value of the best position Gbest, and update Gbest if it is better than the fitness value of the best position; (5) calculate the particle's velocity *V*_*i*_ and position *X*_*i*_ by formulas (1) and (2); and (6) if the end condition is not met, go back to (2); otherwise, end.

### 3.3. SVM Algorithm Model Based on PSO Feature Extraction

Most traditional pattern recognition methods need more training samples, and many practical applications have fewer training samples. Therefore, for a small sample set, the best model trained by machine learning does not mean that it has the best prediction ability. Therefore, how to obtain the best prediction model based on small samples has gradually become a hot and difficult point in the research field of pattern recognition. Support vector machine is a classification algorithm, which is based on statistical theory and adopts structural risk minimization criteria. It has strong generalization ability, especially for pattern recognition problems, such as small samples, nonlinear, and high-dimensional numbers. Support vector machine (SVM) was first derived from the linear separable optimal discriminant surface and then developed further. Then, when classifying the space with higher dimensions, the goal of SVM is to find the hyperplane so that each sample has the maximum distance from it. However, when we apply this algorithm to practical projects, we will find that most of the data in practical applications do not have linear separability. At this time, we will take some measures to solve this problem. At present, the most commonly used measures are to introduce relaxation variables and kernel functions, so that the data can be linearly separable by introducing these two models.

When encountering nonlinear problems, we need to introduce the nonlinear function *∂*(•) and then use this function to train the set. *x* is mapped into a high-dimensional space, and the formula is shown in

(3) $$\begin{array}{c} \partial \left(•\right)=\left(a_{1}\left(x\right),a_{2}\left(x\right),\cdots ,a_{N}\left(x\right)\right). \end{array}$$

In the nonlinear case, the hyperplane is shown in

(4) $$\begin{array}{c} x\cdot \partial \left(x\right)+b=0. \end{array}$$

The decision function is shown in

(5) $$\begin{array}{c} f\left(x\right)=\mathrm{sgn}\left[w\cdot \partial \left(x\right)+b\right]. \end{array}$$

At this time, the model of the optimal problem is obtained by introducing relaxation factors *ξ*_*i*_ ≥ 0, and formula (6) is the model of the optimal problem.

(6) $$\begin{array}{c} \min\partial \left(w,\xi \right)=\frac{1}{2}w\cdot w+C\overset{n}{\underset{i=1}{\sum }}\xi_{i}. \end{array}$$

In order to minimize the risk, the constraint conditions to be met are shown in

(7) $$\begin{array}{c} y_{i}\left[a\left(x_{i}\right)\cdot w+b\right]\geq 1-\xi_{i},i=1,2,\cdots ,n,\xi_{i}\geq 0. \end{array}$$

The kernel function introduced in this paper is *K*(*x*_*i*_, *x*_*j*_), and the formula is shown in

(8) $$\begin{array}{c} K\left(x_{i},x_{j}\right)=\left(a\left(x_{i}\right),a\left(x_{j}\right)\right). \end{array}$$

The duality of the optimal hyperplane problem is described as

(9) $$\begin{array}{c} \max W\left(a\right)=\overset{n}{\underset{i=1}{\sum }}a_{i}=\frac{1}{2}\overset{n}{\underset{i,i=1}{\sum }}a_{i}a_{j}y_{i}y_{j}K\left(x_{i}x_{j}\right). \end{array}$$

The corresponding decision function is shown in

(10) $$\begin{array}{c} f\left(x\right)=\mathrm{sgn}\left\{\overset{n}{\underset{i=1}{\sum }}a_{i}y_{i}K\left(x_{i},x\right)+b\right\}. \end{array}$$

From the above formula derivation, it can be seen that the choice of kernel function is very important for SVM classification algorithm, and different kernel functions will have different classification results. At present, the most widely used kernel function in practical engineering is radial basis function, which is a nonlinear mapping method. This method maps the sample space to high-dimensional space, thus transforming it into a linear problem and solving the relationship between class attributes and classes. Therefore, this paper chooses radial basis function with certain advantages.

## 4. Result Analysis and Discussion

The system mainly uses the ECG acquisition circuit and NI myRIO as the data acquisition platform, and carries out software design based on the platform. Through software design with good architecture, the functions of hardware can be fully developed. At the same time, a good software development environment is very helpful to improve the performance and development efficiency of software. The PSO algorithm is used to optimize the error penalty factor *C* and kernel parameter *g* in SVM. The simulation process is shown in Figure 3.

As can be seen from Figure 3, during the optimization process of SVM by PS0 algorithm, the optimal values of two parameters *C* and *G* obtained by calculation are *C* = 5.6541 and *G* = 8.6218, where the number of iterations is 100.  Table 1 shows the recognition rate of psychological stress by PSO-SVM algorithm tested 20 times.

As can be seen from Table 1, the average recognition rate of the PSO-SVM algorithm tested for 20 times is 82.50%, and the recognition rate of each test is over 70%.

Without knowing the mathematical equation underlying input-output mapping relationships, SVM has the advantage of learning and storing a large number of input-output mapping relationships. The weights and thresholds will, however, have a significant impact on the training results for the BP neural network. As a result, the PSO algorithm is used in this research to optimize the SVM's weights and thresholds. PSO-SVM has 150 sets of training sample data and test sample data, similarly. 70 groups of data from low-pressure sample groups and 80 groups from high-pressure sample groups. In order to train the network, 55 sets of low-voltage sample data are extracted, and 15 sets of data are used for testing data in order to assess the network's capacity for classification. In contrast, 65 sets of high-voltage sample data are extracted in order to train the network, and 15 sets of data are used to assess the network's capacity for classification.  Figure 4 depicts the fitness curve of the PSO-optimized BP neural network.

PSO-SVM and improved PSO-SVM simulation results, as well as PSO-BP and improved PSO-BP simulation results, are compared. The modified PSO-SVM algorithm has a recognition rate for pressure that is 90.17% on average, which is higher than the recognition rate of the PSO-SVM algorithm.  Table 2 displays the PSO-BP algorithm's and an upgraded PSO-BP algorithm's recognition rate after 20 tests.

The average recognition rate for the PSO-SVM through *N*-network experiment is 84.50%, as shown in Table 2, whereas the average recognition rate for the upgraded PSO-BP network experiment is 94.83%. The enhanced PSO-SVM has a greater rate of pressure recognition than PSO-SVMk. In this study, the labels for the low-pressure sample category and high-pressure sample category are both set to 1.  Figure 5 illustrates a simulation experiment of the upgraded particle swarm optimization BP network test set and the classification accuracy of the PSO-BP neural network technique.

The classification accuracy of enhanced PSO-optimized BP is 93.33%, that of basic PSO-optimized BP is 86.67%, and that of improved BP is increased by 6.66%, according to the simulation experiment in Figure 5. As a result, the upgraded PSO algorithm's optimization of SVM and neural networks has much higher classification accuracy than that of the basic PSO method, demonstrating the program's strong generalization capabilities.  Figure 6 illustrates a visual comparison of the recognition rates of four algorithms used in this study: PSO-SVM, PSO-BP, enhanced PSO-SVM, and improved PSO-BP.

Figure 6 illustrates this more intuitively, showing that the recognition rate of the enhanced particle swarm optimization classifier is higher than that of the basic particle swarm optimization classifier, that of the enhanced PS0-SVM algorithm for pressure is higher, that of the enhanced PSO-BP algorithm for pressure is more stable, and that of the enhanced PSO-BP algorithm for psychological pressure is higher. Therefore, it is possible to determine the pressure state using HRV.

## 5. Conclusions

This paper examines the background and significance of the topic selection of moral education penetration in dance teaching in universities, the review of the literature on this subject, the theoretical underpinnings of moral education penetration in dance teaching in universities, and the problems that currently exist in the process of moral education penetration in dance teaching. Since the inception of modern dance thinking, the idea and practice of teaching rhythm have been developed. It delivers not just a fresh approach to instruction but also a universal truth about the core of dance. It is both a rational step away from traditional dance schooling and a return to it. With the development of body rhythm, people have realized that in order to learn dance, one must first experience and learn body rhythm. This will not only help students to understand the true meaning of dance, but it will also help them to improve their sense of body rhythm and coordination, enhance their artistic sensibility and expressiveness, and help them to open their imagination and creativity. In order to identify and assess the psychological state of the human body, this paper proposes to use HRV signals. Then, using this information, it will analyze and reflect the heart rate variability characteristics of dancing activities and determine how the rules change under various stress conditions. As a result, it can more accurately analyze and identify education psychology and achieve the detection of dance education psychology.

## Figures and Tables

**Figure 1:** Functions of each submodule in online dance teaching system.

**Figure 2:** Architecture of distance learning system.

**Figure 3:** Optimization process of parameters *C* and *G* of SVM by PSO.

**Figure 4:** PSO optimizes the fitness curve of SVM.

**Figure 5:** PSO-SVM algorithm and improved PSO-SVM test set accuracy.

**Figure 6:** Recognition rate of pressure by two algorithms.

**Table 1:** Recognition rate of psychological stress by PSO-SVM algorithm.

Test times	1	2	3	4	5	6	7	8	9	10
Recognition rate (%)	78.45	78.49	80.53	90.15	85.26	86.13	90.45	80.66	89.12	91.45
Test times	11	12	13	14	15	16	17	18	19	20
Recognition rate (%)	80.33	94.02	86.22	87.20	82.20	76.13	70.13	73.16	86.13	76.11

**Table 2:** Comparison of recognition rate between PSO-SVM algorithm and PSO-SVM algorithm tested 20 times.

Test times	1	2	3	4	5	6	7	8	9	10
PSO-SVM algorithm Recognition rate	86.34	90.12	83.26	85.12	80.00	79.12	84.34	89.37	75.15	78.33
Improved PSO-SVM algorithm Recognition rate	93.45	96.42	93.41	90.45	97.13	94.12	96.44	93.33	90.66	93.58

## Data Availability

The data used to support the findings of this study are available from the corresponding author upon request.
